# Circ_0005320 promotes oral squamous cell carcinoma tumorigenesis by sponging microRNA-486-3p and microRNA-637

This article has been retracted.

**DOI:** 10.1080/21655979.2021.2009317

**Published:** 2021-12-30

**Authors:** Xiaotao Zheng, Fang Du, Xuepeng Gong, Ping Xu

**Affiliations:** a Department of Stomatology, Weihai Municipal Hospital, Cheeloo College of Medicine, Shandong University, Weihai, Shandong, China; b Department of Hematology and Oncology, No. 988 Hospital of Joint Logistic Support Force of the Chinese People’s Liberation Army, Zhengzhou, Henan, China; c Imaging Department, PLA Air Force 986 Hospital, Xi’an, Shaanxi, China; d Department of Stomatology, The General Hospital of Western Theater Command, Chengdu, Sichuan, China

**Keywords:** Circ_0005320, miR-486-3p, miR-637, oral squamous cell carcinoma, proliferation, apoptosis

## Abstract

Circ_0005320 was found to be elevated in oral squamous cell carcinoma (OSCC) and accelerated OSCC progression. Here, the potential mechanism of circ_0005320 in OSCC tumorigenesis was explored. The quantitative real-time polymerase chain reaction (qRT-PCR) assay was used to detect the expression of circ_0005320, miR-486-3p, and miR-637. In vitro assays were conducted using cell counting kit-8, colony formation, transwell, angiogenesis, and flow cytometry assays. The targeting relationship between microRNA (miR)-486-3p and miR-637 or circ_0005320 was confirmed using the dual-luciferase reporter and RNA immunoprecipitation (RIP) assays. The Janus Kinase 2/Signal Transducer and Activator of Transcription 3 (JAK2/STAT3) pathway-related proteins were analyzed using Western blot. The murine xenograft model was established to perform in vivo assay. Circ_0005320 expression was higher in OSCC tissues and cells. Knockdown of circ_0005320 suppressed OSCC cell growth, migration, invasion, and induced cell apoptosis in vitro, as well as impeded tumor growth in vivo. Mechanistically, miR-486-3p or miR-637 were confirmed to be a target of circ_0005320. Moreover, the inhibitory effects of circ_0005320 silencing on OSCC growth were reversed by the inhibition of miR-486-3p or miR-637. We also found that circ_0005320-miR-486-3p/miR-637 axis mediated the activation of JAK2/STAT3 pathway. This study revealed a novel regulatory network of circ_0005320-miR-486-3p/miR-637 axis in OSCC progression, suggesting that circ_0005320 might be a potential biomarker and therapeutic target for OSCC.

## Introduction

Oral squamous cell carcinoma (OSCC) is the most common type of head and neck cancer with over 300,000 new cases and more than 140,000 deaths each year in the world [1,2]. Current primary treatment for OSCC, surgery with adjuvant radiation or chemoradiation, has achieved advancement. Nevertheless, the 5-year survival duration of OSCC patients has not made significant progress with approximately 50% for 30 years [3]. Therefore, a comprehensive understanding of the molecular mechanism of OSCC pathogenesis is critically necessary.

Recently, circular RNAs (circRNAs) have been identified to be implicated in the physiological and pathological processes of diseases [4,5], especially in cancers [6]. CircRNAs are a class of endogenous non-coding RNAs with covalently closed-loop structures that lack 5ʹ caps or 3ʹ poly(A) tails; thus, they are resistant to the degradation by RNA exonuclease [7]. In addition, circRNAs are also characterized by high stability, high conservation between species and tissue specificity [8]. Recently, increasing researches suggested that circRNAs are frequently dysregulated in cancers and act as oncogenes or tumor suppressors to participate in the progression of multiple malignancies by regulating cell biological processes, such as proliferation, survival, and metastasis [9–11]. Thus, circRNAs may be the promising diagnostic and therapeutic candidates in cancers. Circ_0005320 is a novel circRNA, which arose from its parental gene Septin-9 (SEPT9). It was found to be up-regulated in oral mucosal melanoma (OMM) and might regulate the metastatic and tumorigenesis of OMM [12]. Moreover, a recent study showed an increase in circ_0005320 in OSCC, and elevation of circ_0005320 accelerated OSCC cell survival, invasion, and migration by miR-1225/Protein Kinase N2 axis. However, large-scale identifications of circ_0005320 in the tumorigenesis of OSCC are not yet reported [13].

Herein, we assumed circ_0005320 acted as an oncogenic molecule in OSCC progression via functioning as a sponge for microRNA (miRNA/miR). This study aimed to investigate the action and potential molecular mechanisms of circ_0005320 in OSCC progression, which may suggest a novel insight into the development of efficient therapeutics for OSCC patients.

## Materials and methods

### Human tissue samples

OSCC tissues and paired non-cancerous tissues (as a control) were collected from 33 OSCC patients who underwent surgical resection at Weihai Municipal Hospital. All cases were newly diagnosed by histopathology and did not receive any preoperative treatment. All samples were stored at −80°C until used. Ethical approval for this study was granted by the Weihai Municipal Hospital, according to the Declaration of Helsinki, and written informed consent was collected from each enrolled individual.

### Cell culture

Human OSCC cell lines (CAL27, HSC-2, and SCC25) and human oral keratinocyte (HOK) cells were purchased from BeNa Culture Collection (BNCC, Beijing, China), and then incubated in 5% CO_2_ atmosphere at 37°C using Dulbecco’s modified Eagle’s medium (DMEM, Invitrogen, Carlsbad, CA, USA) containing 10% fetal bovine serum (FBS) and 1% penicillin/streptomycin, both obtained from Invitrogen.

### Quantitative real-time polymerase chain reaction (qRT-PCR)

The RNA Subcellular Isolation Kit (Active Motif, Carlsbad, CA) was used to perform the extraction of nuclear and cytoplasmic RNA in line with the manufacturer’s instruction. Total RNA was extracted from tissues and cells using TRIzol reagent (Invitrogen). The detection of circRNA was undertaken at 37°C for 15 min through the treatment with RNase R (3 U/mg, Invitrogen). A total of 1 μg RNA was reverse-transcribed into complementary DNAs (cDNAs) using PrimeScript RT reagent Kit (Takara Bio Inc, Kusatsu, Japan). qRT-PCR was then carried out using the SYBR® Select Master Mix (Takara). The U6 or glyceraldehyde-3-phosphate dehydrogenase (GAPDH) was used as an endogenous control gene and the expression of gene was detected using the 2^−ΔΔCt^ method. The primer sequences were listed as follows:

circ_0005320: F 5ʹ-CTGTGGCTGAGGCTACACC-3ʹ, R 5ʹ-ACAGTGGCTCGGAGTAGGG-3ʹ;

SEPT9: F 5ʹ-TTCGGCTACGTGGGGATTG-3ʹ, R 5ʹ-CTGCCCGACCACCATGATG-3ʹ;

miR-486-3p: F 5ʹ-GGCAGCTCAGTACAGGATAAA-3ʹ, R 5ʹ-CGGGGCAGCUCAGUACAGGAU-3ʹ;

miR-637: F 5ʹ-ACACTCCAGCTGGGACTGGGGGCTTTCGGGCT-3ʹ, R 5ʹ-CAGTGCAGGGTCCGAGGTAT-3ʹ;

GAPDH: F 5ʹ-CCCACATGGCCTCCAAGGAGTA-3ʹ, R 5ʹ-GTGTACATGGCAACTGTGAGGAGG-3ʹ;

U6: F 5ʹ-CTCGCTTCGGCAGCACA-3ʹ, R 5ʹ-AACGCTTCACGAATTTGCGT-3ʹ.

### Transient transfection

Oligonucleotide miR-486-3p mimics (miR-486-3p, sense 5ʹ-CGGGGCAGCUCAGU ACAGGAU-3ʹ, antisense, 5ʹ-CCUGUACUGAGCUGCCCGUU-3ʹ), inhibitors (anti-miR-486-3p, 5ʹ-GCCCCGUCGAGUCAUGUCCUA-3ʹ), miR-637 mimics (miR-637, sense 5ʹ-ACUGGGGGCUUUCGGGCUCUGCGU-3ʹ, antisense 5ʹ-GCAGAGCCCG AAAGCCCCCAGUUU-3ʹ), inhibitors (anti-miR-637, 5ʹ-ACGCAGAGCCCGAAAG CCCCCAGU-3ʹ), circ_0005320-specific small interfering RNA (siRNA) (si-circ_0005320, 5ʹ-GCCAGGAGGCTTGAAAAGATdtdt-3ʹ), and their respective negative control oligonucleotides (miR-NC sense 5ʹ-UUCUCCGAACGUGUCACGU TT-3ʹ, antisense 5ʹ-ACGUGACACGUUCGGAGAATT-3ʹ; anti-miR-con 5ʹ-CAGUA CAUUGGUUCUGCAA-3, and si-NC, 5ʹ-TTCTCCGAACGTGTCACGT-3ʹ) were purchased from GenePharma (Shanghai, China). Then, CAL27 and SCC25 cells were seeded onto 6-well plates, and transfection was conducted using Lipofectamine 2000 (Invitrogen).

### Cell counting kit-8 (CCK-8) assay

The transfected CAL27 and SCC25 cells were seeded in 96-well plates (3 × 10^4^ cells/well). At 0 h, 24 h, 48 h, and 72 h, per well was added with 10 μL CCK-8 solution (Beyotime, Shanghai, China) and continued to incubate for 2 h. The absorbance was examined at 450 nm using a microplate spectrophotometer (Bio-Rad, Hercules, CA, USA).

### Colony formation assay

After assigned transfection, CAL27 and SCC25 cells (1 × 10^3^ cells/well) were plated at 6-well plates and maintained at 37°C with 5% CO_2_ for 12 days. Culture medium was replaced every 3 days. Finally, the colonies with cluster size of over 50 cells were counted after staining (100×).

### Transwell assay

Transwell chambers (8 mm pore size, Costar, Cambridge, MA, USA) were used to investigate cell invasion and migration. For the transwell migration assay, transfected CAL27 and SCC25 cells in serum-free medium were placed in the upper chamber containing the non-coated membrane. For the invasion assay, transfected CAL27 and SCC25 cells were in serum-free medium were placed in the upper chamber with matrigel-coated membrane (BD Biosciences, San Jose, CA, USA). The lower chambers were loaded with DMEM containing 10% FBS. 24 h later, the migrated and invaded cells in the lower chambers were stained using crystal violet, and cells in five randomly selected fields were imaged and counted (200×).

### Tube formation assay

Pre-chilled 96-well plates were coated with 200 μL Matrigel (BD Biosciences) per well and incubated to polymerize for 30 min at 37°C. After the assigned transfection, the conditioned medium of CAL27 and SCC25 cells were collected, and then HUVECs were seeded onto matrigel plates at a density of 3 × 10^4^ cells/mL with conditioned medium and cultured for 18 h with 5% CO2 at 37°C. The number of branches at random from each culture was counted using a microscope (Olympus DP71 microscope; Olympus, Tokyo, Japan).

### Flow cytometer

Cell cycle was evaluated with flow cytometry after 48 h transfection. Transfected CAL27 and SCC25 cells were trypsinized and rinsed with pre-cold D-Hanks. After centrifugation, the supernatant was discarded, and cells were fixed in 70% cold ethanol for 1 h. Fixed cells were rinsed with cold D-Hanks and stained with 50 mg/mL of propidium iodide (PI) (BD Biosciences). Finally, the FACScan flow cytometer (BD Biosciences) was employed to analyze cell cycle distribution.

CAL27 and SCC25 cells, followed assigned transfection, were trypsinized, rinsed, and then resuspended in 300 μL 1 × binding buffer. Thereafter, the cells were mixed with 5 μL Annexin V-fluorescein Isothiocyanate and 5 μL propidium iodide in the dark at room temperature for 15 min. The apoptotic cells were determined using FACScan flow cytometry (BD Biosciences) within 1 h.

### Dual-luciferase reporter assay

The wild type (WT) or mutant (MUT) 3ʹ untranslated regions (3ʹUTR) sequences of circ_0005320 on miR-486-3p or miR-637 binding regions were separately cloned into pmirGLO luciferase vectors (GeneCreat, Wuhan, China) to generate wild-type pmirGLO-circ_0005320 vectors (circ_0005320 WT) or mutated pmirGLO-circ_0005320 vectors (circ_0005320 MUT). Then, CAL27 and SCC25 cells were co-transfected with 300 ng luciferase vectors and 50 nM miR-486-3p, miR-637, or negative control using Lipofectamine 2000 (Invitrogen). The firefly luciferase activity was evaluated using the dual-luciferase reporter system (GeneCreat) after 24 h transfection.

### RNA immunoprecipitation (RIP) assay

RIP assay was performed using the Magna RNA-Binding Protein Immunoprecipitation Kit (Millipore, Billerica, MA, USA). Briefly, the magnetic beads conjugated with human anti-Argonaute-2 (Ago2) antibody (Millipore) or normal mouse IgG (Abcam, Shanghai, China) were co-transfected into CAL27 and SCC25 cells. The cells were then collected, dissolved in RIP lysis buffer, and then incubated with proteinase K to digest the protein. Finally, the immunoprecipitated RNAs were eluted, purified, and measured using qRT-PCR.

### Western blot

Total proteins were isolated using radioimmunoprecipitation assay buffer (RIPA) (Beyotime) and separated by 10% sodium dodecyl sulfate polyacrylamide gel electrophoresis (SDS-PAGE). Proteins were then transferred onto polyvinylidene difluoride membranes (Millipore) and blocked in 5% skim milk for 1 h. The membranes were incubated with primary antibodies against proliferating cell nuclear antigen (PCNA) (ab29, 1:1000), B-cell lymphoma protein 2 (Bcl-2) (ab692, 1:1000), Bcl-2-associated X (Bax) (ab32503, 1:1000), cleaved caspase 3 (ab32042, 1:5000), total caspase 3 (ab32351, 1:5000), phosphor (p)-STAT3 (Signal Transducer and Activator of Transcription 3) (ab76315, 1:3000), STAT3 (ab119352, 1:5000), p-JAK2 (Janus Kinase 2) (ab195055, 1:2000), JAK2 (ab108596, 1:5000), and GAPDH (ab181602, 1:5000) at 4°C overnight, followed by incubation with corresponding horseradish peroxidase (HRP)-conjugated anti-rabbit IgG secondary antibody (cat. no. AP132P, 1:5000, Millipore) at 37°C for 2 h. The results were analyzed using an enhanced chemiluminescence (ECL) detection system (Beyotime). The primary antibodies were obtained from Abcam.

### Animal experiment

Four- to six-week-old BALB/c nude mice were obtained from Charles River Labs (Beijing, China) and randomly divided into two groups (N = 6 per group). SCC25 cells (3 × 10^6^ cells) stably infected lentivirus-mediated short hairpin RNA targeting circ_0005320 (sh-circ_0005320) or the negative control (sh-NC) (GeneCopoeia, Rockville, MD, USA) was subcutaneously injected into the right flank of nude mice. Tumor size was detected every week to calculate tumor volume. At day 28, the mice were killed, all tumors were stripped, weighed, and divided either for the detection of circ_0005320, miR-486-3p, and miR-637 expression by qRT-PCR or fixed in formalin for Ki67 immunohistochemistry (IHC) staining [14]. The animal experiment was manipulated in line with the protocols permitted by the Ethics Committee of Weihai Municipal Hospital.

### Statistical analysis

Statistical data were expressed as the mean ± standard deviation (SD) and analyzed using GraphPad Prism 7 software (GraphPad, San Diego, CA, USA). Inter-group comparisons were performed using one-way analysis of variance (ANOVA) with Tukey’s test or Student’s *t* test. *P* < 0.05 suggested statistical significance.

## Results

This study aimed to investigate the action and potential molecular mechanisms of circ_0005320 in OSCC progression. Through the in vitro and in vivo assays, we confirmed that circ_0005320 silencing suppressed OSCC cell proliferation, migration, invasion, angiogenesis, and induced cell apoptosis in vitro, as well as hindered tumor growth in nude mice via targeting miR-486-3p/miR-637.

### Circ_0005320 is highly expressed in OSCC tissues and cells

Circ_0005320 was looped and comprised exons 10 and 11 of its parental gene SEPT9, and the junction sequence was validated by Sanger sequencing (Figure 1a). To confirm the stability of circ_0005320, CAL27 and SCC25 cells were treated with or without RNase R; we then found that circ_0005320 could be resistant to the digestion of RNase R, while the level of the linear SEPT9 mRNA was decreased sharply under the RNase R treatment (Figure 1b, c). In addition, subcellular fractionation assay showed that circ_0005320 was prominently localized in the cytoplasm of OSCC cells (Figure 1d, e). All these data indicated that circ_0005320 is a stable circRNA.

**Figure 1.** Circ_0005320 is highly expressed in OSCC tissues and cells. (a) Schematic illustration showing the genomic location of circ_0005320 generated from its host gene SEPT9, and the back-splice junction sequence was validated by Sanger sequencing. (b, c) qRT-PCR analysis of circ_0005320 and linear forms of SEPT9 mRNA expression in CAL27 and SCC25 cells after RNase R treatment or not. (d, e) qRT-PCR indicating the distribution of circ_0005320, GAPDH, and U6 in the cytoplasmic and nuclear fractions of CAL27 and SCC25 cells. (f, g) qRT-PCR analysis of circ_0005320 expression in OSCC tissues and matched normal tissues, as well as in OSCC cells (CAL27, HSC-2, and SCC25) and HOK cells. *P < 0.05.

To understand the role of circ_0005320 in OSCC, the expression profile of circ_0005320 was detected. The qRT-PCR analysis showed that compared with normal tissues and cells (HOK), circ_0005320 expression was higher in OSCC tissues and cells (CAL27, HSC-2, and SCC25) (Figure 1f, g), suggesting that abnormal expression of circ_0005320 was associated with the tumorigenesis of OSCC.

### Circ_0005320 knockdown suppresses OSCC cell growth, migration, invasion, angiogenesis, and induces cell apoptosis

To explore the biological functions of circ_0005320 in OSCC cells, the siRNA targeting circ_0005320 (si-circ_0005320) was designed and transfected into CAL27 and SCC25 cells. As expected, the transfection of si-circ_0005320 significantly reduced circ_0005320 expression in cells, but did not affect the expression of linear SEPT9 (Figure 2a, b). After that, functional experiments were performed. CCK-8 assay suggested that silencing of circ_0005320 inhibited the proliferation of CAL27 and SCC25 cells (Figure 2c, d). The colony formation assay exhibited that the colony formation rates of circ_0005320-decreased CAL27 and SCC25 cells were lower than those in control cells with si-NC (Figure 2e). The results of the transwell assay suggested that cell invasion and migration were attenuated in si-circ_0005320 group relative to si-NC group (Figure 2f, g). In addition, the tube formation assay indicated that compared to the si-NC group, relative numbers of branches formed by HUVECs in si-circ_0005320 group were significantly lower (Figure 2h). Meanwhile, cell cycle was evaluated by flow cytometry. As shown in Figure 2i, circ_0005320 knockdown suppressed cell cycle progression by arresting the CAL27 and SCC25 cells at G0/G1 phase. Furthermore, it was also found that circ_0005320 down-regulation induced apoptosis in CAL27 and SCC25 cells (Figure 2j). Moreover, we also found that the expression levels of PCNA and Bcl-2 were decreased, while the level of Bax was increased in circ_0005320-down-regulated CAL27 and SCC25 cells (Figure 2k, l), and besides that, the ratio of cleaved caspase 3/total caspase 3 was also increased in CAL27 and SCC25 cells after circ_0005320 down-regulation (Figure 2m, n), indicating proliferation inhibition and apoptosis promotion. Taken together, circ_0005320 knockdown repressed OSCC progression by inhibiting cell malignant phenotypes.

**Figure 2.** Circ_0005320 knockdown suppresses OSCC cell growth, migration, invasion and induces cell apoptosis. (a-n) CAL27 and SCC25 cells were transfected with si-circ_0005320 or si-NC. (a, b) Detection of circ_0005320 expression in CAL27 and SCC25 cells using qRT-PCR. (c, d) CCK-8 assay for cell proliferation. (e) Colony formation assay for the colony formation rates of cells. (f, g) Transwell assay for cell migration and invasion. (h) Tube formation assay for cell tube formation ability. (i, j) Flow cytometry for the analysis of cell cycle and apoptosis. (k-n) Western blot analysis of PCNA, Bcl-2, Bax, cleaved caspase 3, and total caspase 3 protein levels in cells. *P < 0.05.

### miR-486-3p or miR-637 is a target of circ_0005320

To investigate the mechanism underlying the promoting effects of circ_0005320 on OSCC, the targeted miRNAs of circ_0005320 were predicted using the circinteractome database. Numerous miRNAs were predicted to have binding site on circ_0005320, and five miRNAs were found to have multiple binding sites on circ_0005320. Among the five miRNAs, miR-486-3p or miR-637 was discovered to be involved in the tumorigenesis in OSCC [15,16]. Thus, we speculated that miR-486-3p or miR-637 might be a target of circ_0005320 in OSCC. The potential binding site between circ_0005320 and miR-486-3p is shown in Figure 3a. We found that miR-486-3p mimic significantly elevated miR-486-3p expression in CAL27 and SCC25 cells (Figure 3b), and then dual-luciferase reporter assay was performed to verify the potential interaction between circ_0005320 and miR-486-3p. The results suggested that miR-486-3p overexpression reduced the luciferase activity of the wild-type circ_0005320 vector but not the mutant one in CAL27 and SCC25 cells (Figure 3c, d). Furthermore, RIP assay indicated that circ_0005320 and miR-486-3p were significantly enriched in Ago2 immunoprecipitates compared to other control RNAs in CAL27 and SCC25 cells (Figure 3e, f). Thus, we verified that circ_0005320 directly targeted miR-486-3p. After that, the expression profile of miR-486-3p was investigated. qRT-PCR analysis showed a marked decrease of miR-486-3p expression level in OSCC tissues and cells (Figure 3g, h), suggesting that miR-486-3p abnormal expression might be related to OSCC tumorigenesis.

**Figure 3.** miR-486-3p or miR-637 is a target of circ_0005320. (a) The potential binding site between circ_0005320 and miR-486-3p. (b) qRT-PCR analysis of miR-486-3p expression in CAL27 and SCC25 cells transfected with miR-486-3p or miR-NC. (c-f) The interaction between circ_0005320 and miR-486-3p was detected by dual-luciferase reporter assay and RIP assay in CAL27 and SCC25 cells. (g, h) qRT-PCR analysis of miR-486-3p expression in OSCC tissues and matched normal tissues, as well as in OSCC cells (CAL27, HSC-2, and SCC25) and HOK cells. (i) The potential binding site between circ_0005320 and miR-637. (j) qRT-PCR analysis of miR-637 expression in CAL27 and SCC25 cells transfected with miR-637 or miR-NC. (k-n) The interaction between circ_0005320 and miR-637 was detected by dual-luciferase reporter assay and RIP assay in CAL27 and SCC25 cells. (o, p) qRT-PCR analysis of miR-637 expression in OSCC tissues and matched normal tissues, as well as in OSCC cells (CAL27, HSC-2, and SCC25) and HOK cells. *P < 0.05.

According to the prediction of the circinteractome database, it was also found the potential binding sites of miR-637 on circ_0005320 (Figure 3i). After confirming the transfection efficiency of miR-637 mimic (Figure 3j), dual-luciferase reporter assay showed that the luciferase activity in CAL27 and SCC25 cells co-transfected with miR-637 and circ_0005320 WT was markedly declined (Figure 3k, l). RIP assay suggested that the Ago2 antibody was able to pull down both endogenous circ_0005320 and miR-637 in CAL27 and SCC25 cells, further validating their binding potential (Figure 3m, n). Meanwhile, the expression of miR-637 was also found to be down-regulated in OSCC tissues and cells (Figure 3o, p), further suggesting the potential involvement of miR-637 in OSCC tumorigenesis.

### Circ_0005320 knockdown suppresses OSCC cell malignant phenotypes by regulating miR-486-3p

We then elucidated whether miR-486-3p mediated the effects of circ_0005320 on OSCC cells. It was found that miR-486-3p inhibitor (anti-miR-486-3p) significantly reduced miR-486-3p expression in CAL27 and SCC25 cells (Figure 4a), and then si-circ_0005320 and anti-miR-486-3p were co-transfected into CAL27 and SCC25 cells, as expected, anti-miR-486-3p introduction attenuated circ_0005320 knockdown-induced increase of miR-486-3p expression in CAL27 and SCC25 cells (Figure 4b, c). After that, a rescue assay was conducted. The results exhibited that miR-486-3p inhibitor reversed circ_0005320 knockdown-evoked inhibition of cell proliferation (Figure 4d, e), colony formation ability (Figure 4f), migration (Figure 4g), invasion (Figure 4h), tube formation ability (Figure 4i), and cell cycle (Figure 4j, k), as well as promotion of cell apoptosis (Figure 4l) in CAL27 and SCC25 cells. Moreover, inhibition of miR-486-3p in circ_0005320-down-regulated CAL27 and SCC25 cells resulted in an increase in PCNA and Bcl-2 expression and decrease in Bax expression and cleaved caspase 3/total caspase 3 ratio (Figure 4m-p). Altogether, circ_0005320 knockdown impeded OSCC cell malignant phenotypes by regulating miR-486-3p.

**Figure 4.** Circ_0005320 knockdown suppresses OSCC cell malignant phenotypes by regulating miR-486-3p. (a) qRT-PCR analysis of miR-486-3p expression in CAL27 and SCC25 cells transfected with anti-miR-486-3p or anti-miR-con. (b-p) CAL27 and SCC25 cells were transfected with si-NC, si-circ_0005320, si-circ_0005320 + anti-miR-con, or si-circ_0005320 + anti-miR-486-3p. (b, c) qRT-PCR analysis of miR-486-3p expression in CAL27 and SCC25 cells. (d, e) CCK-8 assay for cell proliferation. (f) Colony formation assay for the colony formation rates of cells. (g, h) Transwell assay for cell migration and invasion. (i) Tube formation assay for cell tube formation ability. (j-l) Flow cytometry for the analysis of cell cycle and apoptosis. (m-p) Western blot analysis of PCNA, Bcl-2, Bax, cleaved caspase 3, and total caspase 3 protein levels in cells. *P < 0.05.

### Circ_0005320 knockdown suppresses OSCC cell malignant phenotypes by regulating miR-637

Subsequently, we examined the potential involvement of miR-637 in the action of circ_0005320 on OSCC cells. qRT-PCR analysis showed that miR-637 inhibitor reduced miR-637 expression in CAL27 and SCC25 cells (Figure 5a). Then, CAL27 and SCC25 cells were co-transfected with si-circ_0005320 and anti-miR-637, and we found that miR-637 expression was increased by si-circ_0005320, which was reduced by the introduction of miR-637 inhibitor (Figure 5b, c). After that, we performed a rescue assay. miR-637 inhibitor led to the decrease in cell proliferation rate (Figure 5d, e) and colony formation rate (Figure 5f), the reduction of cell migration, invasion (Figure 5g, h) and tube formation abilities (Figure 5i), the delay of cell cycle (Figure 5j, k) and the increase in cell apoptotic rate (Figure 5l) in circ_0005320-decreased CAL27 and SCC25 cells. Moreover, the decreases of PCNA and Bcl-2 expression levels and increases of Bax expression and cleaved caspase 3/total caspase 3 ratio caused by circ_0005320 silencing were abolished in response to miR-637 inhibitor (Figure 5m-p) in CAL27 and SCC25 cells. Overall, circ_0005320/miR-637 axis was responsible for OSCC tumorigenesis.

**Figure 5.** Circ_0005320 knockdown suppresses OSCC cell malignant phenotypes by regulating miR-637. (a) qRT-PCR analysis of miR-637 expression in CAL27 and SCC25 cells transfected with anti-miR-637 or anti-miR-con. (b-p) CAL27 and SCC25 cells were transfected with si-NC, si-circ_0005320, si-circ_0005320 + anti-miR-con, or si-circ_0005320 + anti-miR-637. (b, c) qRT-PCR analysis of miR-486-3p expression in CAL27 and SCC25 cells. (d, e) CCK-8 assay for cell proliferation. (f) Colony formation assay for the colony formation rates of cells. (g, h) Transwell assay for cell migration and invasion. (i) Tube formation assay for cell tube formation ability. (j-l) Flow cytometry for the analysis of cell cycle and apoptosis. (m-p) Western blot analysis of PCNA, Bcl-2, Bax, cleaved caspase 3, and total caspase 3 protein levels in cells. *P < 0.05.

### Circ_0005320/miR-486-3p or circ_0005320/miR-637 axis mediates the activation of JAK2/STAT3 pathway

The activation of the JAK2/STAT3 pathway has been reported to play critical roles in several oncogenic processes including proliferation, differentiation, and angiogenesis in several types of cancers [17,18]. Thus, whether the JAK2/STAT3 pathway is involved in the effects of circ_0005320/miR-486-3p or miR-637 axis on the OSCC progression was further investigated. Western blot analysis showed that circ_0005320 knockdown resulted in the repression of JAK2 and STAT3 phosphorylation, which were attenuated by the introduction of miR-486-3p inhibitor (Figure 6a, b) or miR-637 inhibitor (Figure 6c, d) in CAL27 and SCC25 cells. Therefore, we demonstrated that circ_0005320/miR-486-3p or circ_0005320/miR-637 axis could activate JAK2/STAT3 pathway on OSCC cells.

**Figure 6.** Circ_0005320/miR-486-3p or circ_0005320/miR-637 axis mediates the activation of JAK2/STAT3 pathway. (a-d) Western blot analysis of p-JAK2, JAK2, p-STAT3, and STAT3 expression levels in CAL27 and SCC25 cells. *P < 0.05.

### *Circ_0005320 knockdown hinders OSCC tumor growth* in vivo

Furthermore, a subcutaneous xenograft model was established to validate the biological function of circ_0005320 in vivo. Consistent with the results in vitro, circ_0005320 knockdown significantly reduced the tumor volume (Figure 7a) and tumor weight (Figure 7b, c) compared with those in the control group. Moreover, qRT-PCR analysis showed the level of circ_0005320 was decreased, while the levels of miR-486-3p and miR-637 were increased in the xenograft tissues of sh-circ_0005320 groups (Figure 7d). In addition, IHC staining revealed that circ_0005320 knockdown led to the reduction of Ki67 protein in xenograft tissues (Figure 7e). Collectively, our findings indicated that circ_0005320 knockdown could inhibit OSCC growth in vivo.

**Figure 7.** Circ_0005320 knockdown hinders OSCC tumor growth in vivo. (a) Tumor volumes were measured in the xenograft mouse models. (b) Representative images of the xenograft tumors isolated from two indicated groups. (c) The average tumor weight at day 28 was measured. (d) qRT-PCR analysis of circ_0005320, miR-486-3p, and miR-637 expression in the xenograft tumors of each group. (e) IHC staining for Ki67 in the xenograft tumors of each group. *P < 0.05.

## Discussion

OSCC is usually detected at an advanced stage, and the clinical outcome is less than satisfactory due to the high rates of treatment failure and disease recurrence [19]. It is of great significance to comprehensively understand the molecular mechanisms involved in OSCC growth and metastasis and identify new therapeutic targets. In recent years, aberrant expression of circRNAs has been identified in OSCC, and circRNAs have been exhibited to have roles in the progression of OSCC. For example, Chen et al. found that hsa_circRNA_100290 exerted oncogenic effects to promote OSCC cell survival by regulating cell glycolysis through miR-378a/Glucose transporter 1 (GLUT1) axis [20]. Down-regulation of cirCBCL11B suppressed cell proliferation and migration in vitro via miR-579/LASP1 (LIM and SH3 Protein 1) axis in OSCC [21]. CircRNA_0000140 was demonstrated to serve as a tumor suppressor by repressing tumor metastasis and growth through the inhibition of Hippo signaling pathway via miR-31/Large Tumor Suppressor Kinase 2 (LATS2) axis [22]. In the present study, we found that circ_0005320 was markedly elevated in OSCC tissues and cells. Functional studies revealed that silencing of circ_0005320 could lead to the reduction in cell survival and mobility, the inhibition of angiogenesis, and the increase in cell apoptosis in vitro. Subcutaneous tumor growth was observed in nude mice, and circ_0005320 knockdown also reduced tumor growth in vivo, indicating the clinical relevance of circ_0005320 in OSCC. These results uncovered the tumor-promoter role of circ_0005320 in OSCC, and we believed that circ_0005320 siRNA might be a therapeutic approach for OSCC.

It is known that the biological effects of circRNAs are largely dependent on their subcellular localization. Increasing evidence has manifested that circRNAs located in the cytoplasm can act as competing endogenous RNAs (ceRNAs) to abrogate the repression of miRNAs on target mRNAs at the posttranscriptional level [23,24]. Through the use of subcellular fractionation assay, circ_0005320 was discovered to be mainly located in the cytoplasm, suggesting its potential for serving as miRNA sponges. After that, bioinformatics analysis predicted that circ_0005320 contained putative binding sites of miR-486-3p and miR-637, and subsequent assays verified their interactions. miRNAs are small non-coding single-stranded RNA molecules of ~23 nucleotides. Previous researches have reported that miRNAs are powerful modulators of complex biological processes, including cell growth, apoptosis, metastasis, and metabolism [25], Additionally, it was also revealed that aberrant miRNA expression was associated with the progression of many types of cancer [26,27], including OSCC [28]. miR-486-3p and miR-637 are well-recognized tumor suppressors [29,30] and have been uncovered to impede OSCC tumorigenesis [15,16]. In this study, a decreased miR-486-3p or miR-637 expression was observed in OSCC. Furthermore, miR-486-3p inhibition or miR-637 silencing attenuated the anticancer caused by circ_0005320 knockdown on OSCC. Thus, a significant reciprocal repression feedback loop circ_0005320-miR-486-3p/miR-637 was identified in OSCC.

JAK2/STAT3 signal pathway is a classical intracellular signal transduction pathway, involved in many pathophysiological processes, including cell proliferation, differentiation, inflammation, as well as pain formation [17,31]. Recently, further evidence has suggested that the activation of the JAK2/STAT3 pathway plays an oncogenic role in the progression of OSCC [32,33]. Thus, whether circ_0005320-miR-486-3p/miR-637 axis regulated OSCC progression in a JAK2/STAT3 pathway-dependent manner was investigated. The results showed that circ_0005320 knockdown led to a repression of JAK2 and STAT3 phosphorylation, which were rescued by the inhibition of miR-486-3p or miR-637; thus, we confirmed that circ_0005320-miR-486-3p/miR-637 axis mediated the activation of AK2/STAT3 pathway.

## Conclusion

In conclusion, this work first demonstrated circ_0005320 as an oncogene in OSCC progression by promoting cell growth and metastasis through sequestering miR-486-3p/miR-637. These findings suggest the clinical value of circ_0005320 siRNA in OSCC treatment.

## Highlight

- Circ_0005320 was highly expressed in OSCC tissues and cells.
- Knockdown of circ_0005320 suppressed OSCC cell proliferation, migration, invasion, angiogenesis, and induced cell apoptosis in vitro.
- Circ_0005320 directly interacted with miR-486-3p and miR-637.
- The inhibitory effects of circ_0005320 knockdown on OSCC cells were reversed by the inhibitor of miR-486-3p or miR-637.
- Silencing of circ_0005320 suppressed tumor growth in vivo.
- Circ_0005320-miR-486-3p/miR-637 could mediate the activation of JAK2/STAT3 pathway.

## References

[1] Chi AC, Day TA, Neville BW. Oral cavity and oropharyngeal squamous cell carcinoma–an update. CA Cancer J Clin. 2015;65(5):401–421.2621571210.3322/caac.21293

[2] Sasahira T, Kirita T. Hallmarks of cancer-related newly prognostic factors of oral squamous cell carcinoma. Int J Mol Sci. 2018;19(8):2413.10.3390/ijms19082413PMC612156830115834

[3] Warnakulasuriya S. Global epidemiology of oral and oropharyngeal cancer. Oral Oncol. 2009;45(4–5):309–316.1880440110.1016/j.oraloncology.2008.06.002

[4] Marques-Rocha JL, Samblas M, Milagro FI, et al. Noncoding RNAs, cytokines, and inflammation-related diseases. FASEB J. 2015;29(9):3595–3611.2606585710.1096/fj.14-260323

[5] Altesha MA, Ni T, Khan A, et al. Circular RNA in cardiovascular disease. J Cell Physiol. 2019;234(5):5588–5600.3034189410.1002/jcp.27384

[6] Patop IL, Kadener S. circRNAs in cancer. Curr Opin Genet Dev. 2018;48:121–127.2924506410.1016/j.gde.2017.11.007PMC5877416

[7] Geng Y, Jiang J, Wu C. Function and clinical significance of circRNAs in solid tumors. J Hematol Oncol. 2018;11(1):98.3006446310.1186/s13045-018-0643-zPMC6069963

[8] Yang R, Xing L, Zheng X, et al. The circRNA circAGFG1 acts as a sponge of miR-195-5p to promote triple-negative breast cancer progression through regulating CCNE1 expression. Mol Cancer. 2019;18(1):4.3062170010.1186/s12943-018-0933-7PMC6325825

[9] Chen T, Yang Y. [Role of circular RNA in diagnosis, development and durg resistance of lung cancer]. Zhongguo Fei Ai Za Zhi. 2019;22(8):532–536.3145114510.3779/j.issn.1009-3419.2019.08.09PMC6717870

[10] Feng Y, Wang Q, Shi C, et al. Does circular RNA exert significant effects in ovarian cancer? Crit Rev Eukaryot Gene Expr. 2019;29(2):161–170.3167927110.1615/CritRevEukaryotGeneExpr.2019025941

[11] Bi W, Huang J, Nie C, et al. CircRNA circRNA_102171 promotes papillary thyroid cancer progression through modulating CTNNBIP1-dependent activation of β-catenin pathway. J Exp Clin Cancer Res. 2018;37(1):275.3042481610.1186/s13046-018-0936-7PMC6234664

[12] Ju H, Zhang L, Mao L, et al. Altered expression pattern of circular RNAs in metastatic oral mucosal melanoma. Am J Cancer Res. 2018;8(9):1788–1800.30323971PMC6176177

[13] Ai Y, Tang Z, Zou C, et al. circ_SEPT9, a newly identified circular RNA, promotes oral squamous cell carcinoma progression through miR-1225/PKN2 axis. J Cell Mol Med. 2020;24(22):13266–13277.3309070510.1111/jcmm.15943PMC7701517

[14] Liang Y, Song X, Li Y, et al. LncRNA BCRT1 promotes breast cancer progression by targeting miR-1303/PTBP3 axis. Mol Cancer. 2020;19(1):85.3238489310.1186/s12943-020-01206-5PMC7206728

[15] Chou ST, Peng HY, Mo KC, et al. MicroRNA-486-3p functions as a tumor suppressor in oral cancer by targeting DDR1. J Exp Clin Cancer Res. 2019;38(1):281.3125319210.1186/s13046-019-1283-zPMC6599238

[16] Huang W, Cao J, Peng X. LINC01234 facilitates growth and invasiveness of oral squamous cell carcinoma through regulating the miR-637/NUPR1 axis. Biomed Pharmacother. 2019;120:109507.3159012510.1016/j.biopha.2019.109507

[17] Yu H, Jove R. The STATs of cancer–new molecular targets come of age. Nat Rev Cancer. 2004;4(2):97–105.1496430710.1038/nrc1275

[18] Kong H, Zhang Q, Zeng Y, et al. Prognostic significance of STAT3/phosphorylated-STAT3 in tumor: a meta-analysis of literatures. Int J Clin Exp Med. 2015;8(6):8525–8539.26309504PMC4537978

[19] Ou D, Blanchard P, El Khoury C, et al. Induction chemotherapy with docetaxel, cisplatin and fluorouracil followed by concurrent chemoradiotherapy or chemoradiotherapy alone in locally advanced non-endemic nasopharyngeal carcinoma. Oral Oncol. 2016;62:114–121.2786536410.1016/j.oraloncology.2016.10.011

[20] Chen X, Yu J, Tian H, et al. Circle RNA hsa_circRNA_100290 serves as a ceRNA for miR-378a to regulate oral squamous cell carcinoma cells growth via Glucose transporter-1 (GLUT1) and glycolysis. J Cell Physiol. 2019;234(11):19130–19140.3118748810.1002/jcp.28692

[21] Zeng W, Guo M, Yao L, et al. Circular RNA hsa_circ_0033144 (CircBCL11B) regulates oral squamous cell carcinoma progression via the miR-579/LASP1 axis. Bioengineered. 2021;12(1):4111–4122.3428880410.1080/21655979.2021.1953214PMC8806526

[22] Peng QS, Cheng YN, Zhang WB, et al. circRNA_0000140 suppresses oral squamous cell carcinoma growth and metastasis by targeting miR-31 to inhibit Hippo signaling pathway. Cell Death Dis. 2020;11(2):112.3204194210.1038/s41419-020-2273-yPMC7010827

[23] Du WW, Zhang C, Yang W, et al. Identifying and characterizing circRNA-protein interaction. Theranostics. 2017;7(17):4183–4191.2915881810.7150/thno.21299PMC5695005

[24] Hansen TB, Jensen TI, Clausen BH, et al. Natural RNA circles function as efficient microRNA sponges. Nature. 2013;495(7441):384–388.2344634610.1038/nature11993

[25] Bartel DP. MicroRNAs: genomics, biogenesis, mechanism, and function. Cell. 2004;116(2):281–297.1474443810.1016/s0092-8674(04)00045-5

[26] Yanaihara N, Caplen N, Bowman E, et al. Unique microRNA molecular profiles in lung cancer diagnosis and prognosis. Cancer Cell. 2006;9(3):189–198.1653070310.1016/j.ccr.2006.01.025

[27] Zhang Y, Liu H, Li W, et al. CircRNA_100269 is downregulated in gastric cancer and suppresses tumor cell growth by targeting miR-630. Aging (Albany NY). 2017;9(6):1585–1594.2865754110.18632/aging.101254PMC5509457

[28] Sun C, Li J. Expression of MiRNA-137 in oral squamous cell carcinoma and its clinical significance. J buon. 2018;23(1):167–172.29552778

[29] Yang H, Huang Y, He J, et al. MiR-486-3p inhibits the proliferation, migration and invasion of retinoblastoma cells by targeting ECM1. Biosci Rep. 2020;40(6).10.1042/BSR20200392PMC727391632401301

[30] Du YM, Wang YB. MiR-637 inhibits proliferation and invasion of hepatoma cells by targeted degradation of AKT1. Eur Rev Med Pharmacol Sci. 2019;23(2):567–575.3072016410.26355/eurrev_201901_16869

[31] Li CD, Zhao JY, Chen JL, et al. Mechanism of the JAK2/STAT3-CAV-1-NR2B signaling pathway in painful diabetic neuropathy. Endocrine. 2019;64(1):55–66.3083058510.1007/s12020-019-01880-6PMC6453875

[32] Oh HN, Oh KB, Lee MH, et al. JAK2 regulation by licochalcone H inhibits the cell growth and induces apoptosis in oral squamous cell carcinoma. Phytomedicine. 2019;52:60–69.3059991310.1016/j.phymed.2018.09.180

[33] Jiang X, Huang Z, Sun X, et al. CCL18-NIR1 promotes oral cancer cell growth and metastasis by activating the JAK2/STAT3 signaling pathway. BMC Cancer. 2020;20(1):632.3264109310.1186/s12885-020-07073-zPMC7346480

